# Long Delays and Missed Opportunities in Diagnosing Smear-Positive Pulmonary Tuberculosis in Kampala, Uganda: A Cross-Sectional Study

**DOI:** 10.1371/journal.pone.0014459

**Published:** 2010-12-29

**Authors:** Ibrahim Sendagire, Maarten Schim Van der Loeff, Mesach Mubiru, Joseph Konde-Lule, Frank Cobelens

**Affiliations:** 1 Public Health Department, Kampala City Council, Kampala, Uganda; 2 Center for Poverty Related Communicable Diseases, Academic Medical Centre, Amsterdam, The Netherlands; 3 Centre for Infection and Immunity Amsterdam, Academic Medical Centre, Amsterdam, The Netherlands; 4 Department of Research, Cluster Infectious Diseases, Municipal Health Services, Amsterdam, The Netherlands; 5 School of Public Health, Makerere University College of Health Sciences, Kampala, Uganda; 6 Department of Research, Amsterdam Institute for Global Health and Development, Amsterdam, The Netherlands; University of Stellenbosch, South Africa

## Abstract

**Background:**

Early detection and treatment of tuberculosis cases are the hallmark of successful tuberculosis control. We conducted a cross-sectional study at public primary health facilities in Kampala city, Uganda to quantify diagnostic delay among pulmonary tuberculosis (PTB) patients, assess associated factors, and describe trajectories of patients' health care seeking.

**Methodology/Principal Findings:**

Semi-structured interviews with new smear-positive PTB patients (≥15 years) registered for treatment. Between April 2007 and April 2008, 253 patients were studied. The median total delay was 8 weeks (IQR 4–12), median patient delay was 4 weeks (inter-quartile range [IQR] 1–8) and median health service delay was 4 weeks (IQR 2–8). Long total delay (>14 weeks) was observed for 61/253 (24.1%) of patients, long health service delay (>6 weeks) for 71/242 (29.3%) and long patient delay (>8 weeks) for 47/242 (19.4%). Patients who knew that TB was curable were less likely to have long total delay (adjusted Odds Ratio [aOR] 0.28; 95%CI 0.11–0.73) and long patient delay (aOR 0.36; 95%CI 0.13–0.97). Being female (aOR 1.98; 95%CI 1.06–3.71), staying for more than 5 years at current residence (aOR 2.24 95%CI 1.18–4.27) and having been tested for HIV before (aOR 3.72; 95%CI 1.42–9.75) was associated with long health service delay. Health service delay contributed 50% of the total delay. Ninety-one percent (231) of patients had visited one or more health care providers before they were diagnosed, for an average (median) of 4 visits (range 1–30). All but four patients had systemic symptoms by the time the diagnosis of TB was made.

**Conclusions/Significance:**

Diagnostic delay among tuberculosis patients in Kampala is common and long. This reflects patients waiting too long before seeking care and health services waiting until systemic symptoms are present before examining sputum smears; this results in missed opportunities for diagnosis.

## Introduction

Despite improvements in many aspects of tuberculosis control, delayed diagnosis of tuberculosis still remains a big challenge in many countries. The burden of disease attributable to TB is still huge [1]. Early detection and effective treatment of cases are the hallmark of any successful tuberculosis control programme [2]. Identification and cure of infectious TB cases is recommended as the most cost-effective control measure [3].

Delayed diagnosis results in more extensive disease [4], complications and increased mortality [5]. Delayed diagnosis and treatment lead to prolonged infectiousness [6]. The costs arising from the delay in diagnosing TB are substantial and may worsen the economic situation of patients and their families [7].

Studies in Africa have shown that diagnostic delay is a major problem, with a median duration varying from 8 to 16 weeks across settings [8]–[11]. Diagnostic delay can be divided into patient and health system delay, reflecting the time until consultation is sought and the time between first consultation and final diagnosis of TB, respectively [9]–[11].

In Uganda, one of the high-burden TB countries, TB control is challenged by an estimated low case detection rate of only 51% [1]. Few data have been published about diagnostic delay in Uganda. Limited data exist on where patients go for help when they have TB symptoms and where patients might be diagnosed earlier. A recent study found a median total delay to treatment of 12 weeks among 231 smear-positive pulmonary tuberculosis (PTB) patients newly diagnosed at the national referral hospital in Kampala [12].

We studied diagnostic delay among smear-positive PTB patients registered for treatment at primary care clinics in Kampala city, Uganda. Our aims were to quantify diagnostic delay, to assess factors associated with this delay, to describe trajectories of patients' movements through the health system, and to determine the proportion of patients with systemic symptoms at the time of diagnosis.

## Methods

### Study setting

A questionnaire survey was conducted among newly diagnosed smear-positive PTB patients at Kiruddu, Kisenyi and Kiswa health centres between April 2007 and April 2008. These centres are among ten public primary health care facilities operated by Kampala City Council (KCC), and offer outpatient services including smear microscopy and TB treatment. These centres were purposefully chosen considering geographical representation. Kiruddu health centre is located in a semi-rural residential area. Kisenyi health centre is located in the middle of a densely populated low-income area. Kiswa health centre is located in an industrial area of the city. The health centres often face challenges of heavy patient load, understaffing and periodic stock-outs of various commodities. Health services at these centres are free of charge [13].

Patients seen at these clinics are normally walk-ins from home and referrals from various practitioners within or outside Kampala. Diagnosis of PTB is by direct smear microscopy. The standard procedure of diagnosing PTB in Uganda at the time was that all patients with cough for two weeks or longer were requested to submit three sputum samples. The first and third are on the spot, while the second is an early morning sample. PTB is treated according to the National Tuberculosis and Leprosy Control Programme (NTLP) guidelines. TB treatment is usually initiated on the same day the diagnosis is confirmed. The standard 8 months treatment regimen (2RHZE/6EH) is used as first line treatment.

### Study design

All patients aged ≥15 years diagnosed with sputum smear-positive PTB and registered for treatment at the three KCC clinics within six weeks prior to the day of the interview, were consecutively recruited. Interviews were by semi-structured questionnaire. Patient TB treatment cards were used to ascertain the date treatment was started; this information was confirmed by checking the clinic TB register.

Exclusion criteria were: previous history of tuberculosis treatment for ≥1 month; residence outside Kampala district or beyond a 16 km radius from the city centre. Information was collected on the duration of symptoms in number of weeks before seeking medical care, the date of patient's first consultation with a health care provider and the dates of consultations with subsequent providers, if any, until TB treatment was initiated.

We specifically asked for symptoms frequently associated with PTB: cough, hemoptysis, night sweats, chest pain, fever and patient-reported loss of weight. Data were also collected on socio-demographic characteristics, presence of other medical conditions and knowledge about TB. Patients were requested to tell what causes TB, how TB can be transmitted from one person to another, how one can prevent contracting TB (open questions for each) and whether or not TB can completely be cured (Yes/No/Don't know response).

### Definitions

Patient delay was defined as the time in weeks from the onset of cough to a first consultation with any health care provider, health service delay as the time in weeks from the first consultation to initiation of treatment, and total delay as the sum of both. Definitions of long delays were based on programme-relevant as well as data-driven considerations. Aiming to have 15–30% of patients in the “long delay” category for statistical reasons, we defined long total, long patient and long health service delays as delays of more than 14, 8 and 6 weeks respectively.

Cough was chosen to define delay because it is the most sensitive symptom for smear-positive TB and used as the symptom of entry for TB diagnosis in the NTLP. We defined systemic symptoms as any patient-reported fever, weight loss or night sweats.

### Analysis

Data were collected and double entered into ASP.NET screens, and stored in a customised database based on MS SQL (Microsoft, Seattle, WA, USA). Statistical analyses were carried out using Stata v10 (StataCorp, College Station, TX, USA).

Asset scores from the Health Nutrition and Population country reports were used to assess patient's household wealth [14]. The total score was then divided into tertiles: lower, medium and higher household wealth categories.

In three separate multivariable logistic regression models we analysed associations between a range of explanatory variables and total, patient and health service delay. We entered age (in four categories), sex, type of health care provider first visited and travel cost to the clinic in the models and any other variables if they showed association in the univariate analysis at p<0.20. We included variables in the final model if they contributed to the model likelihood at p<0.05 or confounded the association with any of the other variables in the model.

For a more in-depth analysis of health services' delays, all patients were grouped according to the first provider they visited with their initial symptoms. Within each group, they were sub-grouped by the second provider visited (i.e. in time), then sub-grouped by the 3rd provider, and so on. We retrospectively constructed trajectories by which patients had passed through the health system before being diagnosed with TB.

### Ethical review

This study received ethical approval from the Medical Ethics Committees of Makerere University School of Public Health and the Academic Medical Centre, Amsterdam. Written informed consent was obtained from all participants.

## Results

### Study population

During the study period 614 patients were registered for TB treatment at the three clinics, of whom 417 (68.0%) had smear-positive TB (figure 1). One hundred sixty four patients did not fit the inclusion criteria or refused; 254 eligible patients were interviewed. One patient did not have cough as one of the presenting symptoms and was excluded from this analysis. Table 1 shows the socio-demographic characteristics of the 253 patients included in the study and 150 patients, ≥15 years with complete data on sex, age and clinic registered for treatment during the recruitment period. There were no significant differences for age and sex among patients included in the analysis and those who were not. However, the proportion of non-inclusions was significantly higher in Kiswa (47%) than in the other two clinics (p<0.005).

**Figure 1:** Flowchart showing the patients included in the analysis of diagnostic delay in Kampala, Uganda 2007-8. Legend: KCC = Kampala City Council, TB = Tuberculosis, PTB = Pulmonary tuberculosis.

**Table 1:** Socio-demographic, clinical and diagnostic characteristics of 403 smear-positive pulmonary tuberculosis patients registered for treatment at three Kampala City Clinics, Uganda 2007-8.

Characteristic	Included in analysis N (%)	Not included in analysis N (%)	p value
	253	150	
**Median age**			
30 years (IQR 25–37)		-	=
**Age group**			0.638
15–24 years	60 (23.7)	37 (24.7)	=
25–34 years	106 (41.9)	54 (36.0)	=
35–44 years	62 (24.5)	44 (29.3)	=
>44 years	25 (9.9)	15 (10.0)	=
**Sex**			0.629
Male	149 (58.9)	92 (61.3)	=
Female	104 (41.1)	58 (38.7)	=
**Marital status**			
Single	89 (35.2)	-	=
Married/cohabiting	108 (42.7)	-	=
Divorced/separated/widowed	56 (22.1)	-	=
**Employment status**			
Unemployed	84 (33.2)	-	=
Employed	169 (66.8)	-	=
**City clinic**			0.005
Kiruddu	44 (17.4)	16 (10.7)	=
Kisenyi	136 (53.8)	68 (45.3)	=
Kiswa	73 (28.9)	66 (44.0)	=

The median age of the patients was 30 years (IQR 25–37); 149 (58.9%) were male. Forty four patients (17.4%) were recruited from Kiruddu, 136 (53.8%) from Kisenyi and 73 (28.9%) from Kiswa. These patients were not significantly different in terms of sex (p = 0.954) and age (p = 0.985).

Sixty-five (25.7%) patients registered for treatment at the KCC clinics had been diagnosed at the referral hospital. The remaining 188 (74.3%) patients were both diagnosed and registered for treatment at the KCC clinics. These two groups of patients did not differ significantly by sex (p = 0.211) nor by KCC clinic where they registered (p = 0.494). The median age of patients diagnosed at the referral hospital was 28 years (IQR 25–33), which was lower than of those diagnosed at the city clinics, 32 years (IQR 25–38.5), (p = 0.010).

In addition to cough, patients presented at the time of diagnosis with the following symptoms: loss of weight 220 (87.0%), fever 196 (77.5%), night sweats 189 (74.7%), chest pain 187 (73.9%), haemoptysis 62 (24.5%), and others 21 (8.3%); 249 (98.4%) had at least one systemic symptom.

### Duration of and risk factors for delay

Median total delay was 8 weeks (IQR 4–12). For 61 patients (24.1%) it was longer than 14 weeks (long total delay). Sex, age, cost of transport and first healthcare provider were not significantly associated with long total delay. After adjusting for these variables, patients who knew that TB was curable (adjusted Odds Ratio [aOR] 0.28; 95% CI 0.11–0.73) were significantly less likely to have long total delay (table 2). Long total delay was not associated with education level, marital status, employment status, household wealth, distance of residence from the health centre, type of health facility, or daily intake of alcohol.

**Table 2:** Long total delay and predictor variables of 253 smear-positive pulmonary tuberculosis patients registered for treatment at three Kampala City clinics, Uganda 2007-8.

	Had long total delay		Univariable analysis		Multivariable analysis		
	Yes	No					
	N = 61	N = 192	OR	95%CI	aOR	95%CI	P
**Age**							
15–24 years	10 (16.7)	50 (83.3)	1	-	1	-	0.399
25–34 years	29 (27.4)	77 (72.6)	1.88	0.84–4.20	1.96	0.83–4.62	-
35–44 years	15 (24.2)	47 (75.8)	1.60	0.65–3.90	1.63	0.62–4.28	-
>44 years	7 (28.0)	18 (72.0)	1.94	0.64–5.89	2.28	0.68–7.65	-
**Sex**							
Male	30 (20.1)	119 (79.9)	1	-	1	-	0.079
Female	31 (29.8)	73 (70.2)	1.68	0.94–3.01	1.76	0.94–3.32	-
**Cost of one way journey to health centre in Uganda shillings**							
0–500	36 (27.3)	96 (72.7)	1	-	1	-	0.617
501–1000	14 (18.4)	62 (81.6)	0.60	0.30–1.21	0.71	0.34–1.51	-
1001–1500	6 (20.7)	23 (79.3)	0.70	0.26–1.85	0.58	0.19–1.77	-
1501–20,000	5 (31.3)	11 (68.7)	1.21	0.39–3.73	1.22	0.37–4.07	-
**First provider visited** *							
KCC clinic	9 (33.3)	18 (66.7)	1	-	1	-	0.829
Hospital	4 (25.0)	12 (75.0)	0.67	0.17–2.67	0.41	0.09–1.82	-
Pharmacy/drugshop	12 (25.5)	35 (74.5)	0.69	0.24–1.93	0.79	0.26–2.39	-
Private doctor	12 (26.1)	35 (73.9)	0.71	0.25–1.99	0.89	0.29–2.73	-
Private clinic – other	18 (19.8)	73 (80.2)	0.47	0.18–1.23	0.63	0.22–1.76	-
Traditional healer	3 (25.0)	9 (75.0)	0.67	0.14–3.09	0.78	0.15–3.96	-
**Patient knows TB can be cured**							
No	12 (48.0)	13 (52.0)	1	-	1	-	0.010
Yes	49 (21.5)	179 (78.5)	0.30	0.13–0.69	0.28	0.11–0.73	-

**Legend**

* =  Data available for only 239;

KCC  =  Kampala City Council;

OR =  Odds ratio;

aOR =  adjusted odds ratio;

CI =  Confidence interval;

TB =  tuberculosis.

Complete data on patient and health service delay were available for 242 patients. Median patient delay was 4 weeks (IQR 1–8). Patient delay constituted 50% of the total delay; 47 patients (19%) had long patient delay. Sex, age, cost of transport and first healthcare provider were not significantly associated with long patient delay. Patients who knew that TB was curable (aOR 0.36; 95% CI 0.13–0.97) were significantly less likely to have long patient delay after adjusting for the above variables in the multivariable analysis (table 3).

**Table 3:** Long patient delay and predictor variables of 242 smear-positive pulmonary tuberculosis patients registered for treatment at three Kampala City clinics, Uganda 2007-8.

	Had long patient delay		Univariable analysis		Multivariable analysis		
	Yes	No					
	N = 47	N = 195	OR	95%CI	aOR	95%CI	P
**Age–group**							
15–24 years	13 (22.4)	45 (77.6)	1	-	1	-	0.586
25–34 years	21 (21.0)	79 (79.0)	0.92	0.42–2.01	0.96	0.43–2.17	-
35–44 years	8 (13.3)	52 (86.7)	0.53	0.20–1.40	0.55	0.20–1.49	-
>44 years	5 (20.8)	19 (79.2)	0.91	0.28–2.91	0.95	0.27–3.32	-
**Sex**							
Male	25 (17.6)	117 (82.4)	1	-	1	-	0.566
Female	22 (22.0)	78 (78.0)	1.32	0.70–2.50	1.22	0.62–2.39	-
**Cost of one way journey to health centre in Uganda shillings**							
0–500	27 (20.8)	103 (79.2)	1	-	1	-	0.935
501–1000	12 (17.1)	58 (82.9)	0.79	0.37–1.67	0.85	0.39–1.86	-
1001–1500	5 (19.2)	21 (80.8)	0.91	0.31–2.63	0.72	0.23–2.24	-
1501–20,000	3 (18.8)	13 (81.2)	0.88	0.23–3.31	0.83	0.21–3.35	-
**First provider visited** *							
KCC clinic	6 (22.2)	21 (77.8)	1	-	1	-	0.841
Hospital	4 (25.0)	12 (75.0)	1.17	0.27–4.98	0.95	0.20–4.42	-
Pharmacy/drugshop	8 (17.0)	39 (83.0)	0.72	0.22–2.35	0.81	0.23–2.79	-
Private doctor	12 (26.1)	34 (73.9)	1.24	0.40–3.79	1.39	0.42–4.62	-
Private clinic – other	15 (16)	79 (84)	0.66	0.23–1.92	0.75	0.24–2.35	-
Traditional healer	2 (16.7)	10 (83.3)	0.70	0.12–4.10	0.72	0.12–4.52	-
**Patient knows TB can be cured**							
No	9 (39.1)	14 (60.9)	1	-	1	-	0.050
Yes	38 (17.4)	181 (82.6)	0.33	0.13–0.81	0.36	0.13–0.97	-

**Legend**

* =  Data available for only 239;

KCC  =  Kampala City Council;

OR =  Odds ratio;

aOR =  adjusted odds ratio;

CI =  Confidence interval;

TB =  tuberculosis.

Median health service delay was 4 weeks (IQR 2–8); 71 (29%) patients had long health service delay. Age, cost of transport and first healthcare provider were not significantly associated with long health service delay. Being female (aOR 1.98 95% CI 1.06–3.71), duration of stay at the current residence for more than five years (aOR 2.24 95% CI 1.18–4.27) and having tested for HIV before current TB diagnosis (aOR 3.72 95% CI 1.42–9.75) were significantly associated with long health service delay after adjusting for the above variables in the multivariable analysis (table 4). Household wealth and distance from the health centre were not significantly associated with diagnostic delay.

**Table 4:** Long health service delay and predictor variables of 242 smear-positive pulmonary tuberculosis patients registered for treatment at three Kampala City clinics, Uganda 2007-8.

	Had long HS delay			Univariable analysis		Multivariable analysis		
	Yes		No					
	N = 71		N = 171	OR	95%CI	aOR	95%CI	P
**Age –group**								
15–24 years	11 (19.0)		47 (81.0)	1	-	1	-	0.470
25–34 years	33 (33.0)		67 (67.0)	2.10	0.96–4.58	1.76	0.73–4.24	-
35–44 years	18 (30.0)		42 (70.0)	1.83	0.78–4.32	1.46	0.51–4.13	-
>44 years	9 (37.5)		15 (62.5)	2.56	0.89–7.37	2.47	0.70–8.75	-
**Sex**								
Male	33 (23.2)		109 (76.8)	1	-	1	-	0.031
Female	38 (38.0)		62 (62.0)	2.02	1.15–3.55	1.98	1.06–3.71	-
**Marital status**								
Single	18 (22.0)		64 (78.0)	1	-	1	-	0.462
Married/cohabiting	31 (29.8)		73 (70.2)	1.51	0.77–2.95	1.43	0.65–3.16	-
Divorced/separated/widowed	22 (39.3)		34 (60.7)	2.30	1.09–4.87	1.78	0.70–4.54	-
**Tested for HIV before** *								
No	6 (12.0)		44 (88.0)	1	-	1	-	0.003
Yes	65 (34.0)		126 (66.0)	3.78	1.53–9.34	3.72	1.42–9.75	-
**Cost of one way journey to health centre in Uganda shillings**								
0–500		38 (29.2)	92 (70.8)	1	-	1	-	0.716
501–1000		22 (31.4)	48 (68.6)	1.11	0.59–2.08	1.29	0.64–2.60	-
1001–1500		5 (19.2)	21 (80.8)	0.58	0.20–1.64	0.76	0.25–2.34	-
1501–20,000		6 (37.5)	10 (62.5)	1.45	0.49–4.28	1.53	0.46–5.10	-
**Duration of stay at current residence**								
0–5		35 (25.0)	105 (75.0)	1	-	1	-	0.013
more than 5 years		36 (35.3)	66 (64.7)	1.64	0.94–2.86	2.24	1.18–4.27	-

**Legend**

* =  Data available for only 241;

KCC  =  Kampala City Council;

OR =  Odds ratio;

aOR =  adjusted odds ratio;

CI =  Confidence interval;

TB =  tuberculosis;

HS =  health service.

### Trajectories of patients during contact with the health service

Of the 253 patients, data on first visit to health care provider were unavailable in 11. Among the remaining 242 patients, 231 (95.5%) had visited at least one healthcare provider before the visit at which their TB diagnosis was made. Of the 178 patients diagnosed at the city clinics 9 (5.1%) had been diagnosed during their first visit (figure 2). The remaining 169 patients reported to have consulted on average (median) 1 healthcare provider (range 1–4) in a median of 3 visits (range 1–30).

**Figure 2:** Patients' trajectories through the health system. Legend: The figure shows the health service delay of the patients from the last step of provider before the patient is finally diagnosed with TB. Length of the arrow is equivalent to the length of the delay drawn on scale. Other arrows are not drawn to scale. They just indicate the direction of patient's movement in search of the health care. The width of the arrow represents the number of patients who go from one point to the next. The number in the circles are the total number of patients that start from that point together with those that go through that care provider. In the hospital 2 patients did not experience health service delay. Nine patients did not experience health service delay at the KCC clinics. KCC = Kampala City Council.

The predominant types of provider consulted by these 169 patients in their pre-final visit before a diagnosis of TB was made were private clinics of nurses or midwives for 55 (32.5%), drug shops for 37 (21.9%), and private doctors for 31 (18.3%). Fifteen (8.9%) had already consulted the clinic where they were diagnosed and 14 (8.3%) had consulted a hospital (figure 2).

Of the 64 patients diagnosed at the hospital, 2 (3.1%) had been diagnosed during their first visit. The remaining 62 had consulted on average (median) 2 providers (range 1–3) in a median of 4 visits (range 1–30). Their predominant pre-final visits were to private clinics of nurses or midwives (23; 37.1%), hospitals (13; 21.0%) and private doctors (9; 14.5%), (figure 2).

Table 5 shows the characteristics of patients by the last provider visited before they were eventually diagnosed. The interval between this pre-final visit and the date of diagnosis of TB was shortest for the city clinic where the diagnosis was made (IQR 2–5 weeks) and for private doctors (IQR 2–4 weeks) Although for other providers medians were equal (4 weeks), patients who went to hospital, drug shop or other private provider had long delays in this step. Patients who visited a hospital as the pre-final provider were older than the patients passing through other providers before diagnosis at the city clinics (p = 0.009). Sex and other factors were not associated with delay since the pre-final provider.

**Table 5:** Diagnostic trajectories of tuberculosis patients registered for treatment at three Kampala City clinics, Uganda 2007-8.

Last Clinic of diagnosis	Pre-last provider	n (%)	Median health service delay (IQR)*	Median age (IQR)**	Systemic symptoms
**City Clinics**					
	City clinic	19 (11.2)	3 (2-5)	35.0 (30–40)	18 (94.7%)
	Hospital	14 (8.3)	4 (3-12)	38.0 (29–45)	14 (100.0%)
	Pharmacy/drug shop	41 (24.3)	4 (3-8)	33.0 (29–38)	38 (92.7%)
	Private doctor	31 (18.3)	4 (2-4)	28.0 (22–38)	27 (87.1%)
	Private other	55 (32.5)	4 (2-8)	28.0 (22–37)	49 (89.1%)
**Hospital**					
	Hospital	13 (21%)	4 (3–8)	33.0 (26–24)	13 (100.0%)
	Private other	23 (37.1)	4 (3–8)	26.0 (21–30)	19 (82.6%)
					
Final diagnosis City Clinics (all)		169 (100.0)	4 (2–8)	32.0 (24–38)	155 (91.7%)
Final diagnosis hospital (all)		62 (100.0)	4 (3–8)	28.0 (25–33)	55 (88.7%)
Total in analysis of health service delay		242 (100.0)	4 (2–8)	30.5 (25–38)	210 (86.8%)

**Legend**

Health service delay: from the last provider in the trajectory to start of tuberculosis treatment.

*For those patients finally diagnosed at the city clinics kwallis p-value = 0.088 while those finally diagnosed at hospital kwallis p-value = 1.000.

**For those patients finally diagnosed at the city clinics kwallis p-value = 0.009 while those finally hospital kwallis p-value = 0.029.

Other smaller routes are not shown. Comparisons are only made between the shown groups.

By the time they visited the pre-final provider 155 of 169 (91.7%) patients diagnosed at the city clinics and 55 of the 62 (88.7%) patients diagnosed at the hospital (altogether 90.9%) had systemic symptoms. Altogether 90.9% of patients had systemic symptoms at the time they visited their pre-final provider.

## Discussion

Diagnostic delays in this urban African setting were long. The median total delay was 8 weeks and one quarter (24%) of the patients had delays of more than 14 weeks. This means that a considerable proportion of patients is not diagnosed early and is able to transmit the disease to others for more than 3 months. Half of this delay is due to the delay by the health system. Over 90% of the patients had consulted one or more health care providers before the final diagnosis was made with a median of 4 visits per patient. This suggests that there are many missed opportunities for TB diagnosis in the health system in Kampala.

The patient delays reported in our study are comparable to those reported by other studies from sub-Saharan Africa [8], [9], [12], [15]. The proportion of the total delay that is due to health service delay (50% of the total delay) was somewhat smaller than in an earlier study carried out among patients at the national referral hospital in Kampala (74%). However, it was much higher than that found in Ethiopia (9%) [9], [12]. Health workers in Ethiopia may be more motivated and keen in identifying TB suspects than in Kampala. In addition, there could be more variety in health care providers in the Ugandan health system versus the Ethiopian one, in particular a larger presence of private health care services. In Uganda only public health facilities and a few designated private facilities provide TB treatment; this may increase the health service delay among patients who prefer private providers. The study carried out in the urban referral hospital showed that a sizeable proportion of the patients initially presented to pharmacies or drug shops (40%) [12].

While in our study the type of provider first visited was not associated with long delays, we did observe differences in the health service delay in the final step before the TB diagnosis was made: these were shortest for private doctors and city clinics, suggesting that these tend to refer patients for smear examinations (or advise them to come back), whereas pharmacies and drug shops apparently don't.

Other studies have reported long patient delay to be associated with young age, daily alcohol consumption, subsistence farming, rural residence, distance or cost of travel from home to health institute and low literacy levels [7]–[9], [11], [12]. We found no such associations, probably because of differences in study populations. Ours consisted of urban dwellers. Their literacy levels and levels of awareness are expected to be higher than those residing in the rural areas. Although there are disparities between parts of the city, the health centers in Kampala are fairly accessible from various parts of the city.

We did however find that knowledge that TB can be cured was associated with shorter delays, suggesting that this awareness may take away possible reluctance to be checked for TB. As reported in some other studies female patients experienced more often long health service delay than male patients [6], [16], [17]. It may be that healthcare workers suspect TB less often in women. Health service delays were shorter for patients who had resided at their current residence for less than 5 years suggesting that health care providers have a higher index of suspicion of TB for patients who exhibit alcoholism (which tends to be associated with unstable residence) or are migratory workers. These findings are similar to those reported in a study carried out in rural South African [16].

A surprise finding was that health service delays were longer among patients who had tested for HIV before. Health workers may suspect less TB among patients whose HIV test results are negative. In addition, since we did not include HIV status in the model, this finding may represent confounding by HIV-infected patients having more often low bacillary sputum counts, resulting in the delay of an eventual positive smear.

Why is TB not diagnosed earlier in these patients? Our study suggests a number of reasons. First, patients may initially consult providers who do not suspect TB or find no reason to refer them for smear examination, as seems the case for drug shops and pharmacies. Second, patients may have undergone smear examination but with negative result. This can be because they did not return for a second smear examination (the sensitivity of a single examination being incomplete [18]–[20]), or because they were initially smear-negative. Although we did not ask our study subjects about earlier smear examinations, patients who had earlier visits to the city clinic or hospital may have had earlier smear examinations.

While in the National TB Programme guidelines a cough for ≥2 weeks is considered a reason for smear examination, all but four patients at the time of TB diagnosis and 91% of patients at their pre-final visit had one or more systemic symptoms. Loss of weight, which presents late in the disease process of TB [21], was the second most common symptom (after cough) mentioned by the patients registered for TB treatment at the city clinics.

These data suggest that health care providers wait until the patient is really ill before smear examination is ordered. Indeed, the study carried out in the Kampala urban referral hospital showed that being hospitalized was associated with shorter patient delay [12]. While understandable from the perspective of the city clinics, with a daily load of 100–200 outpatients, shortage of medical and laboratory staff, and no means of pre-selecting high risk patients (such as chest X-ray services), this delay in detecting TB cases for patients already in contact with the health system is a threat to tuberculosis control efforts.

Less than 5% of TB suspects were diagnosed during their first visit to a healthcare provider. Similar findings have been reported in a recent study carried out in China another high burden tuberculosis country [22]. Shortening diagnostic delay in Kampala would require better referral, e.g. by pharmacies, and increased awareness of TB among patients and health care providers. It may be difficult to attain a reduction in diagnostic delay without increasing the efficiency of the diagnostic process so that it can be applied in earlier stages of the disease, e.g. by reducing the number of sputum smear examinations or introducing fluorescence microscopy through which the number of slides that can be processed per day can be substantially increased [23], [24], [25].

Our study had limitations. As with most studies of diagnostic delay, study outcomes were obtained retrospectively and relied entirely on patient self-report. Recall bias could have influenced these results. Only pulmonary smear positive patients were included in this study. The delays would possibly be longer if we had included smear negative and extrapulmonary TB patients. The study was carried out in government health facilities in an urban setting, so its findings cannot be generalised to rural settings. The picture could possibly be different if other forms of TB and private health facilities were included.

Our description of the trajectories was based on cough since this is the most objective symptom directly related to the diagnosis of TB by sputum microscopy. If other TB symptoms were considered, the duration of diagnostic delays might have been longer. The fact that the clinics were purposefully selected could limit the representativeness of our study. A large proportion of registered patients was not included in the study at one of the study sites. This mainly reflected patients living outside the study area, or patients visiting the study clinics outside study days. The latter was responsible for the larger proportion not included in Kiswa clinic where we had only 1 study day per week in the early phase of recruitment. Since it is unlikely that the day of presentation is associated with diagnostic delay, we do not think this introduced selection bias.

Another limitation was that we did not include the data on HIV status in the analysis with the reason that for some patients the status could have been established during the workup for TB diagnosis. In this case knowledge of the HIV status by patient and health care worker would not be an exposure variable for our outcome, diagnostic delay. On the other hand, the biological effect of HIV (in accelerating TB disease clinically or making smears more frequently negative) may have impacted as an exposure variable on diagnostic delay.

Finally, we did no formal sample size calculations and the number of patients in our study sample may have been too small to detect some relevant associations between long delays and patient or health care provider characteristics as statistically significant.

### Conclusions

Diagnostic delays in this patient population are unacceptably high. Patients wait long before consulting the health services, and healthcare providers take long before they diagnose TB. TB cases are not identified by the health system until they develop systemic symptoms. Clinicians and drug shop/pharmacy attendants need to be re-trained to have a high index of suspicion for TB when key symptoms are present. Sensitization campaigns in the communities may help reduce the diagnostic delays. Improved case detection methods are also needed to reduce diagnostic delay. Developing a sensitive screening tool that can identify TB cases earlier is desirable.
